The article "Design and Performance Analysis of a Dynamic Magnetic Resonance Imaging-Compatible Device for Triangular Fibrocartilage Complex Injury Diagnosis" was published in 2022. Journal: J Healthc Eng.

# Design and Performance Analysis of a Dynamic Magnetic Resonance Imaging-Compatible Device for Triangular Fibrocartilage Complex Injury Diagnosis

**DOI:** 10.1155/2022/9688441

**Published:** 2022-06-16

**Authors:** Jiayu Fu, Hui Zhang, Kaiqi Wei, Chao Shi, Wei Zong

**Affiliations:** ^1^China University of Mining and Technology, College of Architecture and Design, School of Industrial Design, 1 Daxue Road, Xuzhou, Jiangsu, China; ^2^Xuzhou TCM Hospital Affiliated to Nanjing University of Chinese Medicine, Department of Radiology, 169 Zhongshan South Road, Xuzhou, Jiangsu, China; ^3^Xuzhou TCM Hospital Affiliated to Nanjing University of Chinese Medicine, Department of Orthopedic, 169 Zhongshan South Road, Xuzhou, Jiangsu, China

## Abstract

Pain and injury of the triangular fibrocartilage complex (TFCC) due to overuse or trauma are commonly diagnosed through static MRI scanning, while TFCC is always involved in radial and ulnar deviation of the wrist. To the best of our knowledge, a dynamic MRI diagnostic method and auxiliary tool have not been applied or fully developed in the literature. As such, this study presents the design and evaluation of a dynamic magnetic resonance imaging (MRI) auxiliary tool for TFCC injury diagnosis. First, 3D scanning and Python are used to measure and fit the radial and ulnar deviation trajectories of healthy participants and patients. 3D printing is then used to manufacture the auxiliary tool for dynamic MRI, and dynamic MRI diagnosis is then conducted to explore the clinical effect. The radial and ulnar deviation trajectory is presented as an asymmetric curve without an obvious circular centre, and the results indicate that the designed auxiliary device meets the requirements of the ulnar and radial movements of the human wrist. According to the MRI contrast test results, the image quality score of patients wearing the auxiliary device is higher than for those without. Such devices could assist clinicians in the diagnosis of TFCC damage, and our method could not only serve as the reference standard for clinical noninvasive diagnosis but also help in understanding the disease and improving the accuracy of TFCC diagnosis.

## 1. Introduction

The wrist joint is one of the most frequently used joints in our daily life, with ulnar deviation of the wrist joint being one of the most commonly used wrist positions [1, 2]. However, ulnar wrist pain occurs frequently and has been noted in several clinical cases [3, 4]. The triangular fibrocartilage complex (TFCC), which is mainly located between the triangular bone and ulna, is used to buffer interbone wear and impact [5]. The common causes of TFCC damage [6] include violent injuries, such as TFCC tear due to hand support during a fall, and degenerative injuries such as aging injuries or severe TFCC wear due to long-term poor manual handling. These not only cause varying degrees of harm to TFCC but also lead to long-term ulnar wrist pain and sequelae, such as distal radioulnar joint instability [7] and limited normal ulnar and radial wrist rotation [8].

Magnetic resonance imaging (MRI) [9] is a good diagnostic imaging method for TFCC injuries, especially for bone, ligament, and soft tissue imaging [10]. Compared to arthroscopic surgery and computed tomography examination, MRI has the advantages of noninvasiveness, painless, absence of radiation, and rapid diagnosis that does not require hospital bed resources.

In recent years, dynamic magnetic resonance imaging (DMRI) technology has been developed and applied in clinical settings. In addition to having the advantages of MRI, DMRI provides a dynamic observation function for diseased tissue. TFCC damage diagnosis through DMRI with carpal tunnel static magnetic resonance images shows the partial radial output of the patient's wrist joint. Meanwhile, wrist movement [3] during wrist tissue state dynamic observation is useful in determining the coherent relationship between the patients' wrist bones and movement. Furthermore, since the jitter caused by patients' ulnar wrist pain produces artifacts in the diagnosis process and reduces image quality, it is necessary to design an auxiliary device to help patients with their DMRI diagnosis and improve imaging quality.

Currently, the study of TFCC injury assistive device design is at its preliminary stage. As assistive devices should have MRI compatibility [11], which is applied in a strong magnetic field environment (1.5 T–3 T), the auxiliary human–machine coordination equipment has special material requirements. In this study, 3D scanning technology and trajectory fitting were combined with actual material and processing technology. An auxiliary device was designed and developed to assist patients with their wrist movement [12, 13], providing a more accurate and reliable MRI basis for clinicians.

## 2. Materials and Methods

### 2.1. Participants

The participants with normal wrist function included 19 Chinese subjects (12 men and 7 women, age: 18–26, hand length: 172–188 mm, hand width: 79–87 mm, and forearm length: 221–238 mm). All participants confirmed that they had no prior hand, wrist, or forearm medical/surgical history and no recent pain/injury in those areas. Each participant read and signed a laboratory certification form.

In addition, one participant with abnormal wrist function admitted to a local hospital for medical treatment with TFCC damage diagnosis was selected. The patient signed an informed consent form noting that she voluntarily participated in the experiment. The patient was guided by the clinician to complete the experiment to avoid secondary injuries/illnesses.

### 2.2. Apparatus

A Creaform HandyScan 300 handheld 3D scanner (scanning accuracy: 0.03 mm, scanning volume accuracy: 0.020 mm + 0.015 mm/m, scanning resolution: 0.05 PMM, and scanning measurement rate: 480,000 measurements per second) was used. The human body models of the forearm, wrist, and palm of the participants were scanned. A Dell laptop (processor: Intel(R) Core(TM)i7-6700QM CPU @ 2.60 GHz; operating memory: 8 GB; hard disk: Seagate 1 TB; graphics card: Intel(R) HD graphics 530, capacity 4160 MB; display: Dell 17-inch display; operating system: Windows 10 64-bit) was used to run the scanning software and store the scanned mannequin records.

We used several 3D scanning reflective points (outer 6 mm, inner 3 mm) to assist the 3D scanner imaging. A pair of wrist straps was used to fix the forearm position of each participant. A high-precision measuring square was used to correct the 0° position of the wrists of the participants. A palm supporting pallet was used to support the hands and fingers of the participants to avoid experimental errors caused by friction between the hands and fingers as well as the plane angle measurement. A measuring plane angle fixed on the experimental platform was used to determine the points in the plane coordinate system, mark the angle marks, and fix the wrist binding band (Figure 1).

### 2.3. Experimental Design

In this study, the measurement range of the wrist joint is selected to represent the ulnar and radial deviation angles as positive and negative, respectively [14]. The whole range of the test is between a radial deviation of 30° and an ulnar deviation of 40°. The participants were required to perform ulnar or radial deviations every 5°, starting at the 0° (i.e., neutral) position of the wrist [3, 15]. After fitting the point cloud of the target marker, the ulnar and radial deviations of the participants' wrists (with normal wrist function and with TFCC injury) were measured. The trajectory curve was used to guide the design of the TFCC magnetic resonance diagnostic auxiliary device.

The entire experiment was conducted under the guidance of a clinician. Both sets of participants were required to perform ulnar and radial deflection of the wrist on the same horizontal working platform. The participants with TFCC injury were required to complete the experiment within the tolerance range of the condition; thus, they were not required to complete the entire process. To obtain more accurate experimental data and remove experimental interference, the participants were required to expose their palms, wrists, and forearms and fit them on the measuring plane angle of the experimental platform (Figure 2(a)).

Before the experiment, the researchers invited the participants to read and explain the experimental guide to ensure that they had a clear understanding of the purpose of the experiment and that they were willing to complete it according to the guidelines. During the experiment, the participants first sat at the bench and adjusted their sitting position accordingly. The researcher subsequently placed, pasted, or bound the necessary materials and performed the 0° wrist correction using a high-precision plane square (Figure 2(b)). After the correction, the scanning began, and the participants were required to perform ulnar/radial rotation at 5° intervals (Figure 3(a)). After each rotation, they were scanned with a handheld device successively at different ulnar and radial angles (Figure 3(b)).

During the experiment, the researchers obtained the 3D models of the forearm, wrist, and palm of the participants under different ulnar and radial deviation angles through scanning. The function to fit the point cloud coordinates of the target marker was used to obtain the ulnar and radial deviation movement trajectory. The base of the third phalanx was selected as the target marker to characterise wrist movement [16–19].

After the experiment, rehabilitation physiotherapists in Xuzhou Hospital of Traditional Chinese Medicine stretched and relaxed the hand muscles, wrist tissues, and forearm muscles of the participants to relieve their fatigue and discomfort during scanning. The intensity of the relaxation task was minimal, thereby preventing physical and psychological stress to the physical rehabilitation therapist.

### 2.4. Statistical Collection and Processing

In this study, the VXelements 8.0 software was used to scan and record the data. The software has the function of establishing an X–Y–Z reference frame according to the scanning reflective coordinates and extracting the point cloud of the target marker. Therefore, the ulnar and radial deviation trajectory fitting of the wrist joint was performed based on this function.

Python 3.9 was used to perform the function fitting of the ulnar and radial deviation trajectories of the wrist joint. The extracted point cloud coordinates were imported into Python 3.9, and the polyfit algorithm of the NumPy library was used to fit the ulnar and radial deviation movement trajectory of the participant's wrist.

## 3. Results

Figure 4 shows the model of the hand, wrist, and part of the forearm of one of the participants at position 0. The coordinates of the target point (base of the third phalanx) in the model were extracted for motion trajectory fitting.

Figure 5(a) shows the ulnar and radial movement trajectories of the wrist of the participants with normal wrist function, which is presented as an asymmetric curve without an obvious circular centre. The participants with normal wrist function had smoother trajectories and smaller curvatures in the radial deviation of 30°–10°. At a radial deviation of 10° and ulnar deviation of 20°, the curved trajectory with large curvature is obtained. Meanwhile, in the ulnar deviation range of 20°–40°, the trajectory is smooth with a small curvature.

Figure 5(b) shows the ulnar and radial movement trajectories of the participant with TFCC injuries. In comparison with participants with normal wrist function, the ulnar and radial motion trajectories of the participant with TFCC injury were similar to that of the participants with normal wrist function. The trajectories of the TFCC-injured participant in the radial deflection range of 30°–10° are relatively smooth with a small curvature. At a radial deviation of 10° and ulnar deviation of 15°, the trajectory is curved with a large curvature. The participant with TFCC injury did not complete the ulnar deviation movement process due to the pain during ulnar deviation movements. Nonetheless, it can be assumed that the trajectory characteristics of the ulnar and radial deviation movement of the wrist joint for the TFCC-injured participant are similar to those of the participants with normal wrist function.

## 4. Design and Setup of the Device for TFCC DMRI Diagnosis

### 4.1. Design of the Device

In this study, the sizes of the auxiliary devices were designed with reference to the “Chinese Adult Body Size Standard” GB10000-1988. The mannequins at the 5^th^, 50^th^, and 95^th^ percentiles of men and women were selected to record the hand and forearm size data, as given in Table 1.

Due to the relatively old data, there is a big difference between the current human body size data; thus, this study aimed to optimize the human body size related to the design of the auxiliary tools. There is an approximate linear relationship between the static size of various parts of the body and height in normal adults [20]. Human height (*H*) is often used to estimate other human body structures. The human body size ratio of Chinese adults is given in Table 2.

Scholars from Tongji University published a work in 2020 predicting the size of the Chinese human body in 2016 according to the growth law of a Chinese body [21]. Based on the proportional relationship between the size of various parts of the human body and height given in Table 2, the size of the hand and arm data in Table 1 is relatively consistent with that of the current human body.

For the 5^th^ percentile female mannequin, the palm length was calculated to be 166 mm, the palm width was 75 mm, and the forearm length was 211 mm. A male mannequin in the 95^th^ percentile had a palm length of 200 mm, a palm width of 91 mm, and a forearm length of 254 mm. The human body data obtained from these calculations were used as the dimensional boundary conditions for the design of auxiliary tools (Table 3).

According to Figure 4, the wrist joint trajectory curve is not a regular circular arc. Thus, the rotational structure design of the auxiliary device for single axis rotation will significantly change the human body structure with regards to the natural wrist movement. As it is not possible to render the natural condition of patients with TFCC injury, the accuracy of the MRI diagnosis is affected, which increases the risk of misjudgement by clinicians.

Therefore, this study focused on the design of a four-link rotational mechanism [22] as the rotational unit of the auxiliary tools. This mechanism has been widely adapted to human joint movement and can meet the wrist movement trajectory curve obtained by the fitting function above without affecting the ulnar and radial deviation movement results of the patient's wrist. Based on the 5^th^ percentile female and 95^th^ percentile male human body models of the hand and forearm dimension data calculated, the auxiliary device was designed. The minimum contract length of the four-bar linkage should be shorter than the 5^th^ percentile female human body model of the hand and forearm size, whereas the maximum length stretch of the mechanism should be longer than the hand and forearm dimensions of the 95^th^ percentile male mannequin.

### 4.2. Device Setup

The auxiliary tools designed in this study used a 3D modelling software using 3D printing and laser cutting technology. As the TFCC damage MRI accessory operates in a special environment exposed to a strong magnetic field of 1.5 T–3 T for a long time, the moulding material has special requirements, including diamagnetism, an antistatic agent, and insulation. Therefore, acrylic [11] was selected as the main moulding material of the auxiliary tool, and an acrylic bolt was selected as the rotation axis of the four-link mechanism. The overall size of the auxiliary equipment conformed to the requirements of the tube wall size of the magnetic resonance machine and did not affect the magnetic resonance diagnostic test. The prototype design and production are shown in Figure 6.

## 5. Performance Analysis of the Auxiliary Device

### 5.1. Experimental Design of MRI Clinical Evaluation

The participant with TFCC injury described in Section 2 was invited to participate in the auxiliary device design evaluation experiment to image the wrist tissue. MRI was conducted with the participant in a prone position [23] with the trouble-side arm extended, while the rest of the body was held still (Figure 7). The experimental process of the participant with TFCC injury MRI-adjuvant design was used as the test group and that without the designed adjuvant as the control group. Proton density imaging sequence was selected for static imaging in both groups. In addition, the T2-SSH-COR-Dyn sequence was used to acquire the dynamic images of the ulnar and radial deflection of the wrists of the participants in the test group.

### 5.2. Evaluation Criteria and Results Based on Imaging Experts

Figure 8 shows a screenshot of the magnetic resonance diagnosis interface for the selected participant. Blind review evaluation was performed by three radiologists with experience of more than 10 years in magnetic resonance diagnosis. The evaluation indices were set according to the consensus of the experts on magnetic resonance examination [24] and in reference to the five-part image evaluation method [25]. Five of the images had high scores, whereas one had a low score (1, wrist bone is blurred and TFCC is not visible; 2, wrist bone is clear and TFCC can be seen but cannot be analysed and evaluated; 3, wrist bone is clear and TFCC is visible, but the boundary is not clear or there is severe blurred background interference; 4, clear wrist bone, visible TFCC, good contrast; 5, clear wrist bone, clear TFCC, clear expression of tissue relationship, good contrast).

Figure 9(a) shows the MRI scan of the participant with TFCC injury when wearing the accessory designed in this study, with an expert score of 4.67 points.  Figure 9(b) shows the MRI scan from the participant with a TFCC injury that did not wear the auxiliary device, with an expert score of 3.67 points.  Figure 10 shows screenshots of the dynamic film of ulnar and radial deviation of the wrist joint output by the T2-SSH-COR-Dyn sequence for the participant with TFCC injury wearing the auxiliary device.  Figure 11 shows the screenshots of the dynamic magnetic resonance films of the participant with wrist deviation movement at a radial deviation of approximately 10° and ulnar deviation of approximately 5° and 20°. These screenshots were used for the comparative analysis of the multiangle MRI scans of wrist deviation movement.

## 6. Discussion

To avoid interfering with the normal ulnar and radial movement of the human wrist, this study scanned and accurately measured the wrist movement track and range of the participants with normal wrist functions and with TFCC injury to guide the design of an auxiliary device for scanning. Applying the design in which the wrist joints rotate in a single shaft rotation, which is common in existing rehabilitation robots [26, 27], to the designed auxiliary device would result in a large intervention for the partial radial movement of the patient's wrist joint. Furthermore, it influenced the DMRI diagnosis and kinematics correlation between the carpal bone and TFCC cartilage in the patient. Therefore, it is important to design a linkage mechanism that does not interfere with the ulnar and radial rotation of the patient.

In this study, the palm length and width and forearm length of the human body in the stage of emergence were deduced through calculation and applied in the auxiliary design. As the designed four-link movement structure has good scalability, it can meet the wearing requirements of different patients and assist the patient in carrying out the ulnar and radial movement of the wrist joint. Simultaneously, the overall size of the auxiliary tool was limited to 600 × 500 mm to meet the diameter size of the magnetic resonance machine channel. The parts used to support the patient's hand and arm were also designed to be light and easy to install, thereby greatly simplifying the operation of the accessory.

In the process of MRI clinical diagnosis evaluation, as shown in Figure 9, and evaluation by the MRI experts, the traditional static MRI scans obtained by the patient wearing the auxiliary devices designed in this study had high quality with the expert score of 4.67 points. In this image, the bone of the wrist joint is distinct, as were the TFCC, peripheral inflammation, and ulnar ligament. The outline of the bone and tissue and position relationship was clear. In contrast, the quality of MRI scans obtained from patients without the auxiliary device was relatively low, with an expert score of 3.67. Due to the jitter caused by the slight swelling of the patient's wrist tissue in the absence of assistance, the artifacts of the MRI scan reduced the image quality. In this image, the contours of the bone of the wrist joint are fuzzy, the TFCC structure, surrounding inflammation, and contours of the bone and tissue are relatively fuzzy, the ulnar ligament is not visible, and the positional relationship is not clear.

With the assistance of the auxiliary device designed in this study, the DMRI of the ulnar and radial movement of the wrist of the patient with TFCC injury was realised using the T2-SSH-COR-Dyn sequence. In this dynamic process, the clinicians can more intuitively observe the movement and position change relationship of the wrist bone of the patient with TFCC injury during exercise. According to the analysis in Figure 11, the clinician concluded that in the process of ulnar and radial deviation of the wrist joint of this patient, a relatively large displacement occurred between the hook bone and triangular bone and between the triangular bone and ulna. This results in excessive stretching and extrusion of the TFCC for a long time, thereby resulting in degenerative injury to the TFCC and pain. Combining the static MRI scans and patient's self-reported absence of a history of violent injury, the orthopaedist determined that the patient could receive conservative treatment without arthroscopic surgery.

Nonetheless, there are several shortcomings in this study. First, there are only a few samples from participants with their left hand as the dominant hand, and the ulnar and radial movement trajectories of the participants with a dominant left hand are limited. When fitting the ulnar and radial deviation motion trajectories of the wrist joint, we selected the polyfit algorithm of Python 3.9 NumPy library for the fitting operation, which can be further optimised in future research. Additionally, as the auxiliary device required the patient to perform the MRI diagnosis in the prone position rather than in the traditional flat position, the patient is more likely to get tired during the experiment.

## 7. Conclusions

In this study, the wrist motion trajectories and motion ranges of participants with a normal wrist function and a patient with TFCC injury were measured. The results were used to guide the design of dynamic magnetic resonance diagnostic tools for TFCC injury. The trajectory of the ulnar and radial deviations of the human wrist joint studied in this work has addressed the gap mentioned in the current literature. The designed linkage structure of the auxiliary device did not only avoid interference with the ulnar and radial movement of the patient's wrist but also met the working and environmental requirements of dynamic magnetic resonance diagnosis. In addition, the auxiliary device can meet the output quality requirements of static MRI and dynamic magnetic resonance and provide image support and dynamic magnetic resonance video support for clinicians, assisting them in follow-up diagnosis and treatment. Therefore, further designs and studies on the wrist auxiliary device are needed to assist the diagnosis of DMRI and further expand the study sample. Finally, we anticipate that this diagnostic method will become the standard for clinical noninvasive diagnosis of TFCC injury.

## Figures and Tables

**Figure 1:** Experimental material and equipment: (a) HandyScan 300 3D scanner, data cables, measuring square, and 3D scanning reflective points. (b) Experimental platform, plane angle measurement, and palm supporting pallet.

**Figure 2:** Preparation and scanning of the experiment. (a) Participants sitting in front of the test bench and (b) 0° wrist position of the participants corrected using a plane square.

**Figure 3:** (a) Ulnar deviation and radial deviation of the wrist and (b) researcher holding a 3D scanner to scan the palm, wrist, and forearm of the participant.

**Figure 4:** Scan of the generated human model of the palm, wrist, and part of the forearm of a participant and extraction of the coordinates of the target markers. The point indicated by the arrow is the target marking point of the scanning experiment.

**Figure 5:** Ulnar and radial trajectories of the wrist of (a) 19 healthy participants and (b) one patient with TFCC injury (the patient did not complete the entire experiment due to the pain caused during the ulnar and radial trajectory measurement).

**Figure 6:** TFCC dynamic magnetic resonance diagnostic aids: (a) design model and (b) prototype.

**Figure 7:** Dynamic magnetic resonance scan of the wrist joint in the prone position with the assistance of the auxiliary device.

**Figure 8:** Screenshot of the DMRI scan interface of the patient's wrist.

**Figure 9:** MRI scans: (a) test group, where the wrist tissue of the patient using an auxiliary device was clearly expressed and TFCC was visible; (b) control group, where artifacts were generated due to the pain and shaking of the patient, thereby reducing the image quality (arrow pointing in the figure is an artifact).

**Figure 10:** Screenshot of the dynamic magnetic resonance video of the ulnar and radial movements of the patient's wrist.

**Figure 11:** Multiangle comparative analysis of the ulnar deviation motions of the wrist of the patient using MRI: (a) radial deviation motion of approximately 10°, (b) ulnar deviation motion of approximately 5°, and (c) ulnar deviation motion of approximately 20° (arrow points to the necrotic lunate, showing the black area in the image. Distance 1 indicates the change in relative position between the uncinate bone and triangular bone. Distance 2 is the change in the relative position between the triangular bone and ulna).

**Table 1:** Hand and forearm sizes of men and women at the 5^th^, 50^th^, and 95^th^ percentiles obtained from the Chinese adult body size standard GB10000-1988.

Gender		Male			Female		
Percentile		P5	P50	P95	P5	P50	P95
Item	Height (mm)	1583	1678	1775	1484	1570	1659
	Forearm length (mm)	216	237	183	193	213	234
	Hand length (mm)	170	183	196	159	171	183
	Hand breadth (mm)	76	82	89	70	76	82

**Table 2:** Ratio of the hand length, hand width, and forearm length to height in Chinese adults.

Serial number	Item	Male (H)	Female (H)
1	Forearm length	0.14	0.14
2	Hand length	0.11	0.11
3	Hand breadth	0.05	0.05

**Table 3:** Comparison of the human hand length, hand width, and forearm length data at 1988 and 2016.

Gender			Male			Female		
Year	Percentile		P5	P50	P95	P5	P50	P95
1988	Item	Height (mm)	1583	1678	1775	1484	1570	1659
		Forearm length (mm)	216	237	258	193	213	234
		Hand length (mm)	170	183	196	159	171	183
		Hand breadth (mm)	76	82	89	70	76	82

2016	Item	Height (mm)	1613	1713	1815	1508	1606	1700
		Forearm length (mm)	226	240	254	211	225	238
		Hand length (mm)	177	188	200	166	177	187
		Hand breadth (mm)	81	86	91	75	80	85

## Data Availability

The video data and 3D scanning models of participants' hands used to support the findings of this study have not been made available because the protection of patient's privacy as well as restrictions from the third party.
